The article "Analysis and Exploration on the Integration of Mental Health Education into College Physical Education Practice" was published in 2022. Journal: Comput Intell Neurosci.

# Analysis and Exploration on the Integration of Mental Health Education into College Physical Education Practice

**DOI:** 10.1155/2022/5195909

**Published:** 2022-08-21

**Authors:** Wei Zhu, Jinhong Li

**Affiliations:** School of Humanities GuangXi Polytechnic of Construction, NanNing 530007, GuangXi, China

## Abstract

In order to understand the mental health status of contemporary college students, the research team of “College Students' psychological quality training” conducted mental health examination on nearly 6000 Chinese college students from 23 colleges and universities across the country. The results showed that about 16.51% of Chinese college graduates had serious mental health problems. The results of several recent studies on the mental health status of college graduates across the country show that the accuracy rate of mental behavior examination among college graduates across the country is about 16%, and the rate of people with unsound psychology or in a state of mental sub-health is higher, and there has been a psychological poverty group among college students. A large number of educational facts and scientific research have confirmed that sports are one of the most effective ways to promote students' physical and mental development, and it can be said that there is a very close relationship between college sports and the physical and mental health of college graduates. In order to promote the organic combination of college mental health education and college physical education, the research results will be based on in-depth investigation and understanding of the current situation of college students' psychological development under the new situation, and a systematic study of the relationship between college graduates' physical, sports, mental health knowledge, and psychological level. This paper establishes a theoretical model for the organic combination of mental health education and physical education in colleges and universities, and provides specific countermeasures for integrating psychological teaching into college physical education courses, providing a theoretical basis and reference for developing college physical education courses and improving psychological teaching.

## 1. Research Object and Research Method

### 1.1. Research Object

Taking the combination of mental health education and physical teaching in colleges and universities as the research object, adopting the method of random stratified sampling, 50 physical teaching classes in 5 colleges and universities, with a total of 1842 people, were selected as the objects of psychological questionnaire survey and physical fitness test. The number of students who effectively answered the psychological questionnaire and participated in all physical fitness index tests was 1715, including 792 boys and 923 girls.

The article "Analysis and Exploration on the Integration of Mental Health Education into College Physical Education Practice" was published in 2022. Journal: Comput Intell Neurosci.

### 1.2. Research Methods

#### 1.2.1. Questionnaire Survey Method

(1) Self-examination and evaluation form of psychological symptoms: the school has adopted the self-examination and evaluation form of psychological symptoms (SCL-90) to investigate and understand the psychological level of college students. (2) Physical exercise psychology measurement scale: the test scale is divided into 8 subscales with 70 items. The contents are physical exercise psychology, goal attitude, sports awareness, physical exercise habits, sports intention, emotional feelings, sense of behavior control, and subjective standards. (3) Human self-esteem scale: College Students' Physical Self-esteem Scale (PSPP) is a standardized tool to measure individual satisfaction and dissatisfaction with all aspects of their physical health under the background of Chinese traditional culture [1].

#### 1.2.2. Constitution Test Method

According to the content of physical examination and assessment for college students stipulated by the Ministry of Education of China, the six values of the subjects' length, weight, vital capacity, step test, standing long jump, and grip strength were measured, and the subjects were divided into good physical fitness group, excellent group, high pass rate group, and unqualified group.

#### 1.2.3. Expert Consultation Method

On the basis of a psychological questionnaire and physical test, aiming at the problems related to the combination of psychological teaching and college physical education courses in colleges and universities, consulting experts engaged in psychological counseling and teaching in colleges and universities.

#### 1.2.4. Mathematical Statistics Method

The data of psychological questionnaire score and physical fitness test score were input into the computer, and then the two evaluation methods were described and analyzed by Excel and SPSS software, and the grey correlation data were analyzed.

## 2. Correlation Analysis between Mental Health and Physical Condition of College Students

### 2.1. Investigation and Factor Analysis of College Students' Mental Health

#### 2.1.1. The Overall Situation of the Investigation on the Mental Health Status of College Students

The Symptom Self-Rating Scale-SCL90 is one of the most famous mental health test scales in the world, and is currently the most widely used outpatient examination scale for mental disorders and mental illnesses. SCL90 helps us to understand our mental health from ten aspects. SCL-90 score refers to the sum of 90 individual scores, which represents the overall level of personal psychological status. The higher the SCL-90 score, the lower the overall level of physical and psychological illness [2]. On the contrary, the higher the overall level of physical and mental illness. Referring to the relevant standard requirements [3]: SCL-90 scores ≥180 is psychological disease, of which 180 ≤ SCL-90 scores <225 are minor psychological disease, 225 ≤ SCL-90 scores <270 are moderate psychological disease, and SCL-90 scores ≥270 is a severe psychological disease. Any one of the nine factors ≥3 points positive test out of mental health education problems. The preliminary statistical results of SCL-90 showed that 226 people had mild psychological disease, accounting for 13.2% of the total population surveyed; the number of students with moderate psychological disease was 157, accounting for 9.7% of the total number investigated; the number of students with severe psychological disease was about 32, accounting for 1.3% of the total number of the survey; 173 college students scored in at least one factor ≥3 points, so the positive test accuracy of mental health problems in this questionnaire survey was about 10.1%. By itemizing nine factors among all college graduates' mental health problems with mental illness, the authors found that among the symptoms of college graduates' mental health illness, the top three were obsessive-compulsive disorder, interpersonal sensitivity, and paranoia, followed by depression, anxiety, and hostility [4]. The above behaviors can lead to psychological phenomena such as uneasiness, inferiority complex, narrow range of interpersonal communication, being unable to speak with most of the students, and being jealous of the advantages of other students, which can lead to depression, painful thinking, and emotional state; they are unwilling to carry out collective and competitive activities, lose interest in game meaning activities item, and are slow to respond [5].

The article "Analysis and Exploration on the Integration of Mental Health Education into College Physical Education Practice" was published in 2022. Journal: Comput Intell Neurosci.

#### 2.1.2. Analysis on the Characteristics of College Students' Mental Health

A total of 1715 college graduates were surveyed this time, including 792 males and 923 females: male : female = 1 : 1.17, age range from 17 to 25 years old, with an average age of 20.41 ± 3.65 years. There are 1614 Han people and 101 national minority people, with a ratio of 15.98 : 1; there are 1183 college graduates from urban registered permanent residence and 532 college graduates from nonurban registered residence, with a ratio of 2.22 : 1; there are 1263 only child college students and 452 not only child college students. The ratio of the two is 2.79 : 1. In order to study the influence of demographic theoretical characteristics such as gender, national, household registration type, and children's situation on the mental health status of college students, the paper screened out the situation of students' mental health problems under various demographic theoretical characteristic variables and carried out *X*2 test. See Table 1 for the impact of the changes in demographic characteristics on the positive test out of college students' mental health problems.

It can be seen from Table 1 that for the psychological health problems of college graduates caused by gender and race variation, the positive test screening has no significant negative impact (*P* > 0.05), and the two variables of registered residence type and family children have significant negative impact on the incidence of psychological disorders of college students. Through the analysis of the nine factor scores among college students with urban registered residence and nonurban registered residence, one-child and not one-child, it is concluded that the five factors of nonurban registered residence college students in interpersonal sensitivity, tension, obsessive-compulsive disorder, somatization, and depression are more prominent than those of urban registered residence college students (*P* < 0.05); the only child in the five factors of paranoia, depression, interpersonal sensitivity, tension, and obsessive-compulsive disorder are more prominent than the nonurban registered residence college students (*P* < 0.05) (see Table 2). It can be inferred that college students' family situation and life background have a great negative impact on their psychological development.

#### 2.1.3. Comparative Analysis of Mental Health Status of Students in Different Grades

The survey covers four age groups in colleges and universities, including 521 freshmen, 507 sophomores, 435 juniors, and 252 seniors. The ratio of the four is 2.07 : 2.01 : 1.73 : 1. Preliminary statistics show that the percentage of students whose psychological questionnaire scores are lower than or more than 180 in each grade is 25.1%, 23.7%, 21.4%, and 19.5%. The positive rate of psychological problems in each grade was 10.6%, 9.7%, 9.4%, and 10.3%. It can be found that there is no significant difference in the accuracy of positive detection of mental health problems among different grades, and with the increase of age, the overall mental health status of college students is gradually improving [6]. In order to further analyze the mental health status of college graduates of all ages, the paper makes a comparative analysis on the scores of nine mental health factors of college graduates of four ages [7]. The results show that the scores of freshmen in interpersonal relationship, tension, hostility, and fear are higher than those in Table 2; the scores of depression, anxiety, paranoia, and psychosis of the third grade college graduates were stronger than those in Table 2, while the scores of somatization and anxiety symptoms of the fourth grade college graduates were better than those of the second and third year students, but the difference was not statistically significant (*P* > 0. 05) (see Table 3).

The article "Analysis and Exploration on the Integration of Mental Health Education into College Physical Education Practice" was published in 2022. Journal: Comput Intell Neurosci.

### 2.2. Comparative Study on Mental Health Level and Physical Condition of College Students

According to the grading standards for the physical fitness evaluation of college graduates nationwide, the overall physical fitness evaluation, vital capacity weight index score, hand grip strength weight index score, step test score, and standing long jump scores are divided into four grades: excellent, good, qualified, and unqualified groups. The height and weight levels were divided into four grades: healthy body, low weight, obesity and insufficient nutrients. For the convenience of comparison, the healthy people were classified as the excellent group, the low weight people were classified as the better group, and the healthy people with poor nutrients were classified as the failed group. After the online evaluation of the measured six original scores, the evaluation results and grades of six indicators are obtained. According to the physique grading standard, the conclusions in Table 4 are obtained. In terms of the overall assessment grade of physical fitness, 96.97% of the college graduates' physical fitness grade has reached the pass level or above, indicating that the overall physical fitness of contemporary college graduates is good [8]. However, in terms of the specific distribution of the other five indicators, the physical quality development of college graduates is not balanced, and some indicators are generally poor, such as the unqualified rates of standing long jump and lung viability weight indicators, which exceed 44.02% and 24.90%, respectively. This shows that it is imperative to strengthen the reform of physical education teaching and promote the coordinated development of college graduates.

#### 2.2.1. Correlation Analysis between College Students' Mental Health Level and Their Physical Indicators

The comprehensive evaluation of physical health level of college students generally adopts the percentage system. The weight of length standard weight, step test, vital capacity body mass index, standing long jump, hand grip strength, and body mass index in the overall evaluation is 0.15, 0.20, 0.15, 0.30, and 0.20, respectively. In order to check whether there are significant differences among the 6 body indexes of college graduates with various psychological levels, the one-way ANOVA is carried out by taking various physical index scores and psychological levels as factors, respectively. At the same time, descriptive statistics are carried out on various physical index scores of college graduates with various psychological levels. After summarizing, the conclusions described in Table 5 are drawn. It can be seen from Table 5 that there is a difference (Sig<0.05) in the scores of other five physical fitness indicators among college students with mental health level in different regions of the country except for the height standard body mass index no difference (SIG>0.05). If the severity was compared with the healthy group, there were significant differences among the 6 body mass indexes. In comparison with the healthy group and the moderate group, except for the two indexes of health standard weight and step test, there were differences among the other four indexes; compared with the healthy group, the mild group had no significant difference among the other three indexes except for the differences in vital capacity body mass index, standing long jump, and height standard weight score. This shows that the physical condition of college graduates is gradually weakening due to the increase in the degree of psychological disease.

The article "Analysis and Exploration on the Integration of Mental Health Education into College Physical Education Practice" was published in 2022. Journal: Comput Intell Neurosci.

#### 2.2.2. Multiple Comparative Analysis of Students' Psychological Factors and Their Physical Conditions

In order to further analyze which of the 9 mental health factors of college graduates have an important impact on the physical state of college students, this paper takes the student's physical grade as factor A, which is divided into 4 levels, takes the student's psychological factor level as factor B, and divides it into 9 levels of mental health factors according to factor B. All levels of mental health factors of A and B under different physical levels at the intersection were T-scores, which were tested by multi-factor analysis of variance and further Duncan multiple factor comparison test.

It can be seen from Table 6 that the differences among the 9 factors of college students of different physical grades have statistical significance (all *P*'s are 0.0001). Among them, the 9 psychological factor problems of the physical unqualified group are much more prominent than those of the physical excellent groups and good groups, especially the four factor problems of paranoia, somatization, enemy, and psychosis. The 4 factors of interpersonal tension, obsessive-compulsive disorder, paranoia, and anxiety item in the physical qualified group were more prominent than those in the physically good group, and there was no specific statistical significance in the other five factors between the two groups (*P* > 0.05). Compared with the good group, the excellent group had no significant difference in the other six basic factors except interpersonal relationship, anxiety, and paranoia. This shows that interpersonal relationship, tension, and paranoia have a great impact on the physical state of college graduates, the four factors of compulsion, depression, somatization, and hostility have the least impact, while the two factors of fear and psychosis have a relatively small impact on the physical state of college graduates [9]. These results illustrate that multiple physical health factors can affect the physical condition of college students, among which interpersonal relationships have the most significant impact on physical condition. This shows that in order to keep college students in good physical condition, building good interpersonal relationships is crucial.

The article "Analysis and Exploration on the Integration of Mental Health Education into College Physical Education Practice" was published in 2022. Journal: Comput Intell Neurosci.

#### 2.2.3. Correlation Analysis between Students' Mental Health Level and Physical Condition

In the research process of the above big data analysis, the author found that there is a certain degree of common change trend between the physical status of college graduates and their mental health level. In order to study the impact of the six physical indicators on the physical and mental health level of college graduates, the physical status of college graduates and their mental and physical health level are now regarded as the same gray system, analyze the relationship between them [10]. Firstly, the reference series *X*_0_ (K) of the physical and mental health level of college graduates is established, that is, the parent factor; the comparison series of total physical score *X*_1_ (*K*), length standard weight score *X*_2_ (K), vital capacity body weight index score *X*_3_ (), grip strength body mass index score *X*_4_ (*K*), step test score *X*_5_ (*K*), and standing long jump score *X*_6_ (*K*), namely, the sub factors. After the initial value of various technical indicators *K*, the absolute value difference list shall be written first, and the judgment coefficient shall be *P* = 0.5. Then, the correlation coefficient and the correlation degree are calculated according to formulas (1) and (2), respectively.

(1) $$\begin{array}{c} §i^{\left(k\right)}=\frac{\Delta \min+p\cdot \Delta \max}{\Delta \text{oi}\left(k\right)+p\cdot \Delta \max}, \end{array}$$

(2) $$\begin{array}{c} r_{i}=\frac{1}{N}\overset{R}{\underset{k-1}{\sum }}\xi_{i}\left(k\right), \end{array}$$

(§*I* represents the correlation coefficient, *r*_*i*_ is the correlation degree, and greater the *r*_*i*_ is, the closer the relationship is.)The final calculation result is: *r*1 = 0.712; *r*2 = 0.527; *r*3 = 0.643; *r*4 = 0.519; *r*5 = 0.557; and *r*6 = 0.612. According to the correlation degree, the order is *r*1 > *r*3 > *r*6 > *r*5 > *r*2 > *r*4. The grey correlation analysis shows that: first, the physical condition of college students affects the physical and mental health level of college students, and the degree of influence is as follows: overall physical condition, vital capacity body mass index, standing long jump performance, step test score, height standard weight, and grip strength body mass index. Second, there is a close relationship between college students' mental health level and their physical condition, but this relationship is not a one-to-one linear relationship [11]. Thirdly, the synchronous change trend between the mental health level of college students and their physical condition is aimed at the college student group, and whether this correlation degree also exists for different individuals needs to be further studied.

The article "Analysis and Exploration on the Integration of Mental Health Education into College Physical Education Practice" was published in 2022. Journal: Comput Intell Neurosci.

## 3. The Combination of College Students' Mental Health Education and Physical Education

### 3.1. Basic Principles between Mental Health Education and Physical Education Teaching Benefits

#### 3.1.1. Principle of Interactivity

Doing a good job in psychological teaching of college graduates is a systematic project to promote the coordinated development of physical and mental health of college graduates. For educators, it involves not only full-time and part-time psychological teachers, but also psychological teachers of other disciplines, as well as teaching management staff at all levels; from the perspective of psychological teaching objects, all college students are the main body of physical education and psychological teaching [12]. For educators, only by communicating with schools can they understand the psychological needs of college graduates, and only by enhancing internal communication and cooperation among educators can they achieve more effective educational action. As the object of psychology teaching, students' self-needs can be better realized only through continuous interaction with educators. Therefore, in the process of interaction between school physical education and college graduates' psychological teaching, schools should also do a good job in the communication and interaction between physical education teachers, psychological teachers, and school education managers. In addition, we should give full play to the resource advantages of school sports extracurricular activities and actively encourage college students to participate in various social activities, so as to realize the communication between health educators and the educated, so as to maximize the effectiveness of school sports activities and health teaching.

The article "Analysis and Exploration on the Integration of Mental Health Education into College Physical Education Practice" was published in 2022. Journal: Comput Intell Neurosci.

#### 3.1.2. Principle of Subjectivity

Whether it is physical education courses or teaching activities, or psychological teaching, it is finally implemented to the college graduates themselves because the main function of teachers is to improve the knowledge level of college students and guide students to find solutions to problems. The function of teachers can only be influenced by the outside world, and the psychological adjustment and physical development of college students ultimately depend on the internal factors and self-awareness of college graduates. Therefore, in order to realize the comprehensive benefits of college physical education and psychology teaching and promote each other, the most effective method that can be used at present is to promote college students to understand the basic psychological knowledge of systematic science through college psychology teaching. At the same time, college sports teaching and extracurricular activities can promote the healthy development of students' body and mind. In the process of benign interaction, college students can optimize their physical quality and solve their psychological problems more actively.

#### 3.1.3. Activity Principle

Social activities are the process of interaction between human subject and objective world. Human psychological activities reflect the object world, and with the help of activities react on the macro world, the reflected object is further tested and developed. Therefore, activities constitute the material basis for the emergence and development of human psychology and the root of the human mind [13]. People's good psychological quality is produced and developed in the process of activities and communication. The improvement of college graduates' physical fitness and psychological level depends on the active participation of college graduates, and the theoretical teaching of psychological teaching alone cannot complete the task [14]. The principle of activity means that both college students and psychological teachers should carry out rich and diverse recreational and sports activities to cultivate and improve students' good psychological quality in specific practice. Therefore, in the interaction between college physical education and college students' health education, the school should give full play to the basic function of physical activity class, and enable college students to carry out exercise and training in various situations by adopting various sports courses or activities.

#### 3.1.4. Principle of Comprehensiveness

The principle of comprehensiveness means that in the process of psychological teaching, educators should use the concept of system theory to guide their work. From the perspective of learners' hearts, their psychological state is an organic whole. Knowledge, behavior, emotion, intention, and behavior are all closely linked. Psychological processes, social psychological conditions, and personal psychological characteristics affect each other. Social psychological factors and personal physiological reasons also complement each other. Starting from the internal and external interpersonal relationship, we should start with the mutual restriction and coordination between personal physical reasons and external environment, and comprehensively consider and analyze the factors and specific measures of learners' psychological problems. Therefore, educators should start with the overall and overall development concept, establish the “humanized” development concept for college graduates, and pay attention to the harmonious development of college students' morality, intelligence, physique, beauty, as well as knowledge, behavior, will, and behavior; secondly, teachers should timely find and make up for the deficiencies in some aspects of students, comprehensively check and analyze the causes of these deficiencies and put forward measures to promote the harmonious development of all aspects of college students' quality.

The article "Analysis and Exploration on the Integration of Mental Health Education into College Physical Education Practice" was published in 2022. Journal: Comput Intell Neurosci.

### 3.2. Basic Objectives of Interaction between Mental Health Education and Physical Education Teaching Benefits

#### 3.2.1. Meet the Needs of College Students and Promote the Coordinated Development of Body and Mind

The diversity of physical education courses, the wide range of college graduates' interests, and different physical conditions all make college graduates have certain differences in learning enthusiasm, ability, and mental health requirements. Therefore, in the process of mutual promotion between school physical education and psychological teaching, on the one hand, school physical education teachers should give full play to the characteristics, connotation, forms, and means of school physical education teaching according to the psychological characteristics and basic requirements of college graduates, combine psychological guidance and teaching, and do a good job in school physical education, extracurricular physical education teaching activities, and student sports competitions. In order to fully provide college graduates with opportunities to fully display themselves and develop themselves, so as to meet the psychological needs of college graduates at all stages. In addition, university psychology and health teaching staff should teach basic psychological knowledge according to the laws of physical and mental development of college students, and study the methods of using sports methods to regulate students' psychological development, so as to create a good atmosphere for in-depth school sports activities and provide basic psychological knowledge guide. The school teachers who play a leading role must also set an example and act as teachers, edify and influence the college graduates through their noble career, profound knowledge, serious and responsible service attitude, approachable work style, and high serviceability.

The article "Analysis and Exploration on the Integration of Mental Health Education into College Physical Education Practice" was published in 2022. Journal: Comput Intell Neurosci.

#### 3.2.2. Strengthen Awareness and Promote Behavior Coordination

Human willpower is displayed through behavior, and behavior is also dominated by willpower. Healthy individuals' will and action are unified and harmonious. The perfection of individual will power is the consciousness, boldness, firmness, and self-control of individual behavior. The collectivist moral education in school physical education is the main content to promote college students to cultivate good psychological quality, and it is also the main way to cooperate with the rapid and healthy development of college graduates' behavioral ability. In college physical education, on the one hand, teachers should properly introduce games or competitions and other teaching methods into the curriculum, so as to promote students' active participation, enhance college students' sense of group and responsibility, improve group concept, and improve group cohesion. In addition, the teachers also consciously screen and set obstacles with different complexity, and guide the learners to exercise their willpower, strengthen their free will, cultivate good habits of rational behavior, and actively deal with negative interference situations by means of autonomous guidance, autonomous instruction, autonomous service, autonomous detection, autonomous supervision, and autonomous responsibility, maintain psychological balance, and promote the harmony and moderation of social behavior by quickly changing situations. Moderate behavior coordination means that in general, for a person with self-awareness, he always knows what he is doing and why he is doing it, and is always able to predict the process and consequences of activities so that his activities serve specific purposes and conditions.

#### 3.2.3. Maintain a Harmonious Relationship and Shape a Sound Personality

Maintaining harmonious interpersonal relationships is not only the main sign of the physical and mental health of college students, but also the main prerequisite for ensuring physical and mental health. The concrete manifestation of harmonious interpersonal communication is as follows: in academic career, he is willing to get along with colleagues and teachers, has a wide and stable relationship, and has close friends; in interpersonal communication, he can get along well with others with respect, integrity, friendliness, tolerance, and understanding, and has a unique and calm personality. Know others as you know yourself, neither humble nor arrogant; be able to judge others objectively and accurately, learn from others' strengths, make up for myself weaknesses, strictly enforce self-discipline, and be lenient to others. Be able to maintain a harmonious interpersonal relationship with the collective, cooperate well with the others, make concerted efforts with others, and actively help others. Independent and complete personality is gradually established in harmonious interpersonal communication. Ensuring the independence and integrity of personality is the ultimate goal of psychological education. Good personality is marked by all elements of personality structure are free of obvious defects and deviations; have correct self-awareness, we can know ourselves, accept ourselves, and properly evaluate our self-worth; value concept has become the core concept of people with a proactive outlook on life and values that adapt to the direction of social development, and has a high sense of obligation and responsibility. Therefore, in the process of mutual promotion between school sports and psychological teaching, sports teaching should create a harmonious interpersonal relationship environment, and form a healthy personality of college students through sports and psychological teaching.

The article "Analysis and Exploration on the Integration of Mental Health Education into College Physical Education Practice" was published in 2022. Journal: Comput Intell Neurosci.

#### 3.2.4. Maintain Emotional Stability and Build Self-Confidence

A stable and happy mood is an important symbol of physical and mental health [15]. In the mental health people, the positive mood is greater than the depressed mood, while the happy mood is dominant; at the same time, people who are physically and mentally healthy can usually coordinate and manage their emotions and maintain a good mental state. Practice has also proved that people who often play sports can directly experience the spiritual pleasure brought by sports, thus producing a happy spiritual feeling; sports can not only make people open, happy, energetic, and full of vitality, but also adjust their mentality, reduce their loneliness and depression, make people excited and full of vitality, and promote the cultivation of self-confidence. Self-confidence is the basic guarantee for a person to succeed. Sports games make participants often have the joy of success or victory, which will undoubtedly improve a person's confidence. However, because self-confidence can be cultivated and established not only in victory, but also in frustration, the failure of a competition often makes participants discover their own shortcomings and the weak links of the other party, thus strengthening their belief in the winning.

The article "Analysis and Exploration on the Integration of Mental Health Education into College Physical Education Practice" was published in 2022. Journal: Comput Intell Neurosci.

## 4. Operation Strategy of Combining Mental Health Education with Physical Education

### 4.1. Teaching Strategy of Combining Mental Health Education with Physical Education

#### 4.1.1. College Physical Education and Mental Health Education Should Pay Attention to Organic Interaction

Organic interactive education means that when teachers carry out psychological teaching in sports courses or physical education teaching activities, they must pay attention to time and content, that is, physical education teachers must seek a reasonable combination with psychological teaching through the content of psychological teaching in sports courses and the available teaching resources contained therein. But generally speaking, the psychological content integrated into each sports teaching course must be contained in the psychological education materials of the course, which is the content of the school, but it cannot be imposed without the sports course. Therefore, all far-fetched and labeled psychological teaching is neither scientific nor reasonable; therefore, it is not advisable to carry out sports courses simply for the purpose of psychological education. Although there are a lot of psychological education contents in physical education courses, not all teaching contents and at what time can be psychological education, and not every physical education course needs psychological education. The psychological internal infiltration in the classroom teaching of physical education majors lies in freedom and Appropriateness. It is closely linked with the characteristics and specific implementation steps of all college physical education courses, and is organically integrated. Therefore, the first strategy to promote college physical education and college students' psychological education is to let nature take its course and minimize far-fetched interaction.

#### 4.1.2. College Physical Education and Mental Health Education Should Be Moderately Interactive

The so-called “appropriate interaction” means that the interaction between modern sports activities and college students' mental health quality education should be “appropriate and limited.” The “appropriate” means that the duration of mental health quality education should not be too long in a physical education class or physical education activity. Because the goal of implementing the mental health curriculum in the sports curriculum class is “secondary purpose,” and the internal normative education goal of the sports curriculum itself is “main purpose,” so it never the guest robs the place of the host. First, we should pay attention to the level of interaction, that is, the overall goal of interaction should not be too high or too low. Second, we should pay attention to the gradient of interaction, that is, on the basis of understanding the personality psychology and individual differences of college students. We should fully consider the acceptability of college students at all levels and the gradual order among them. Third, we should pay attention to the effectiveness of information interaction, that is, teachers should often collect relevant dynamic information of college students and adjust information interaction strategies in time to seize the opportunity of information interaction.

The article "Analysis and Exploration on the Integration of Mental Health Education into College Physical Education Practice" was published in 2022. Journal: Comput Intell Neurosci.

#### 4.1.3. College Physical Education and Mental Health Education Should Be Flexible and Interactive

The interaction between physical education and psychological teaching is not a static way. From the perspective of curriculum design orientation, the interaction between physical education and psychological teaching is mainly centered on school education, focusing on the cultivation of students' character and promoting students' psychological development; it also focuses on the characteristics of sports, and develops the cultivation of students' character and will according to the physical characteristics of college graduates; it may also help college graduates to solve their psychological difficulties by putting questions as the center and integrating theory with practice; it may also focus on teaching activities, strengthen students' psychological exercise, and cultivate students' excellent psychological quality. In terms of the forms of interaction, there are decentralized and centralized, group and individual, discussion and teaching, etc. From the perspective of the interaction mode of the specific content, there are the emotional transfer method, role-playing method, cognitive correction method, psychological game teaching method, and so on. Under the guidance of various values, different interactive strategies are formed through the flexible use of various interactive forms and modes.

### 4.2. Carefully Arrange the Teaching Contents and Methods, and Strive to Develop the Learning Potential of Physical Education

#### 4.2.1. Mental Health Cognitive Knowledge Education

Carrying out psychological cognitive knowledge teaching for college students, in order to promote college students to form new views on mental health education, and pay attention to protecting and improving physical and mental health, can more effectively prevent the occurrence of various diseases among college students. Therefore, in the school physical education and health teaching, teachers should purposefully explore the knowledge connotation with psychological health teaching value in the school physical education curriculum, fill in some relevant teaching materials, and then use the methods of explanation, exchange, and analysis to achieve the two interactive goals. First, help the students of ordinary colleges and universities to understand and be familiar with the basic mental health knowledge and mental health care knowledge, and make it clear that psychology is the performance of certain mental states in a certain period of time, which is corresponding and has grade differences; second, it is clear that sports is the most reasonable and easy to control way to integrate the mind and body. One of the most important goals of sports teaching and training is to maintain and improve the physical and mental health of learners.

The article "Analysis and Exploration on the Integration of Mental Health Education into College Physical Education Practice" was published in 2022. Journal: Comput Intell Neurosci.

#### 4.2.2. High Quality Psychological Learning Education

The purpose of providing excellent sports psychological learning education is to help college students develop sports learning potential, master scientific sports learning methods and strategies, correct wrong sports learning mentality and behavior habits, and improve the effectiveness of sports learning. Its general connotation includes:

1. Learning motivation education. By setting course goals, creating a good sports environment, attribution teaching, positive feedback, value seeking, etc., mobilize the psychological positive motivation of college students to participate in physical education and exercise. Teachers should adopt successful pedagogy, happy pedagogy, needs-satisfaction method, interest-based teaching method, etc., to cultivate the free will, interest, and hobby of college students to participate in sports, so as to change or enhance college graduates' modern sports teaching and sports mentality, cultivate good sports habits, and establish a benign sports psychological state.
2. Psychological stimulation and regulation teaching. In the classroom teaching of physical education, teachers, according to the changes of college students' psychological activities and behavior, carry out psychological stimulation and exerting suggestive control to make them have a positive, excited and studious psychology, so as to effectively mobilize and cultivate their enthusiasm, initiative and innovative ability in physical education learning. The main ways of implementing psychological stimulation control are trust, expectation, inspiration, evaluation, psychological counseling, etc. The main ways of exerting suggestive control are self, others, expression, authority, mark, example, etc.
3. Develop sports skills. It is generally carried out with the help of normal teaching activities and mental health training. Its basic operating procedures generally include: provision of conditions and implementation requirements; during repeated training, the important goal is to be familiar with society, nature, and consciousness; actively guide and actively create a model for students to imitate; supervise and check to help students solve their wrong habits. Similarly, the general methods of spiritual practice of skill cultivation are representation, self-relaxation, concentration, spiritual suggestion, free will, etc.

The article "Analysis and Exploration on the Integration of Mental Health Education into College Physical Education Practice" was published in 2022. Journal: Comput Intell Neurosci.

#### 4.2.3. Appropriate Emotional Education

Emotional adjustment and emotional development is a process of psychosocial activities with the active human cognition [16]. On the one hand, better emotional education has a positive impact on promoting the development of personal morality and knowledge, and improving the level of personal physical and mental growth. In addition, school sports social activities also have a positive and negative impact on personal emotional adjustment and social emotional play. The school carries out emotional education, which aims to help college students learn to adjust their mentality in a timely manner, enhance their ability to control emotions, develop good social emotional awareness, avoid excessive fluctuations in personal emotions, and avoid mental diseases caused by psychological disorders of college graduates. In the process of mutual promotion between school physical education and students' psychological teaching, we can make use of the different emotions contained in school physical social activities to stimulate people, such as overcoming obstacles, participating in competition, self-control, feeling success, and accepting frustration, so as to make school graduates feel success and frustration, happiness and depression, advantages and disadvantages, fairness and difference, fairness and partiality, reasonable and unreasonable, etc. produce diversified feelings, guide college students to correctly treat these feelings, and reasonably treat their personal life needs. At the same time, it is also necessary to consciously use the methods of perception regulation, body language expression regulation, activity regulation, breathing regulation, attention regulation, suggestion regulation, stimulation regulation, self-venting, psychological attribution regulation, etc. to improve students' happiness.

#### 4.2.4. Strong Will Quality Education

Cultivating students' good spiritual character is the main goal of college students' mental health quality education. Sports teaching in colleges and universities is an important means to cultivate the good spiritual character of college graduates. The reason is that in the process of physical education courses and physical training in colleges and universities, students will always face different psychological problems and obstacles, such as students' fear in the process of sports, as well as the external natural environment, weather, sports equipment, and various other factors. Influence, college graduates can build a strong foundation of spiritual character after constantly overcoming the above problems and obstacles. Cultivating the good spiritual character of college students from the sports teaching in colleges and universities can be mainly carried out from the following aspects: first, physical education teachers should establish the subject consciousness of cultivating students' excellent spiritual character; second, in the process of sports teaching, we should give full play to the incentive effect of collective consciousness and example spirit; third, pay attention to the positive effects of sports skills and training; forth, encourage and guide primary and middle school students culture the spirit to fight against difficulty in physical exercise and sports competitions.

The article "Analysis and Exploration on the Integration of Mental Health Education into College Physical Education Practice" was published in 2022. Journal: Comput Intell Neurosci.

#### 4.2.5. Good Character Education

Personality education plays a key role in student education, because personality is not only closely related to the healthy development of people's ideology and morality and the level of knowledge learning, but also closely related to the healthy development of people's spirit. The research of modern medicine and psychology has proved that personality has a significant impact on the occurrence, healthy development and prognosis of human diseases, especially physical diseases. The reason why personality can have a significant impact on the healthy development of human diseases, especially physical diseases, is that the patient's personality characteristics can not only become the basis for the occurrence of a variety of diseases, but also change the process of the healthy development of a variety of diseases, or determine the performance of the disease more than the pathogenic characteristics of some diseases. Therefore, it is very beneficial to improve the mental health of students and promote the harmonious development of mind and body by striving to cultivate liveliness, joy, openness, and other excellent personalities. Personality teaching is mainly divided into two aspects: one is to cultivate students' excellent personality characteristics; the other is to help students correct wrong personality characteristics. Both can be integrated into a good personality structure.

The article "Analysis and Exploration on the Integration of Mental Health Education into College Physical Education Practice" was published in 2022. Journal: Comput Intell Neurosci.

#### 4.2.6. Interpersonal Relative Guidance

Due to the development of social economy and the improvement of the pace of life, many college students have increasingly no proper social relations, and the feelings between people tend to be indifferent. Sports extracurricular activities are a good form for people to communicate with each other, which can enhance the relationship between people and society. In the process of communication between college physical education and mental health teaching, it is emphasized that the main purpose of interpersonal relationship guidance is to coordinate the same good relationship. College students can build up the relationship between peers, relatives, and friends on the sports field, so as to rebuild the new teaching mode of relationship with college students. With the charm of sports, human beings can break through estrangement and isolation, gather strength in the sports field, and build a peaceful, friendly, and harmonious social interpersonal relationship [17]. Sporting activities do not distinguish between social status, wealth, occupation, and age, so that human beings can run fairly and sincerely for a certain goal, and can rejoice and excite for the game, which can further develop the communication skills of university students and further improve the level of social interpersonal communication.

#### 4.2.7. Cultivation of Competition Awareness and Cooperation Spirit

Fair competition is often a form of motivation to improve one's own achievements. It means that individuals or groups compete fairly with others or other groups in order to achieve better achievements; synergy refers to a social activity in which groups work together, and this synergy is to make this group further compete fairly with other groups. And sports is to guide the whole human social activities in the form of fair competition and rich and colorful connotation. In the whole process of sports, fair competitions are always implemented. Even in general sports games, there is a race to catch up and win. The characteristics of sports competition and cooperation have a very positive significance for cultivating the enterprising spirit of college students, activating personal motivation, improving academic level and efficiency, cultivating lofty aspirations, and establishing good personality. At the same time, they can also more effectively cultivate the group will and team spirit of modern people who are good at working with others in social competition. Therefore, through in-depth development of physical education in colleges and universities, it can more effectively promote college graduates to form good psychological quality required by modern society.

The article "Analysis and Exploration on the Integration of Mental Health Education into College Physical Education Practice" was published in 2022. Journal: Comput Intell Neurosci.

#### 4.2.8. Effective Self-Healing Education

Among the main reasons that have been found to reduce the psychological load of personal life, two reasons are particularly obvious: social support and physical exercise. By taking part in sports, people improve their social interaction and get social help more easily. Relevant scientific research has also confirmed that students' physical exercise can help people relieve depression, pessimism, and other negative mentality, reduce anxiety, thus reducing depression and other psychological diseases, so as to keep people in psychological balance and achieve the goal of physical and mental health development. Games, which belong to the means of sports therapy, are also one of the most basic ways of psychological counseling and treatment for students, especially in group counseling. Moreover, student gymnastics can use different intensity and speed to reduce patients' negative psychological, thus achieving the effect of eliminating psychological diseases. The focus of practice is to guide students and teach learners to use a simple and efficient way to carry out their own mental health testing, formulate a targeted plan for exercise according to their own cognitive status, and implement an independent psychotherapy method that integrates self-practice, self-control, self-test, and self-evaluation.

## 5. Specific Ways of Combining Mental Health Education with Physical Education

### 5.1. Special Psychological Lectures

Extracurricular sports practice social activities play an important role in school teaching. It is not only the main teaching content of extracurricular sports education for school students, but also the main component of campus sports. Moreover, extracurricular sports practice social activities are the most basic way for college students to participate in social activities of physical and mental health education, which can promote the mental health of college students. The school extracurricular modern sports practice social activities are divided into extracurricular sports exercise, extracurricular sports training, extracurricular sports competition, and other main basic aspects. It has played a positive role in extracurricular activities on campus with the advantages of rich form flexibility, rich connotation of social activities, broad space for social activities, and strong popularity of participants. It has created a relatively broad living space for social activities for the comprehensive implementation of quality education and the promotion of the harmonious development of physical and mental health of college students. Carrying out colorful extracurricular sports teaching activities can also effectively cultivate the spirit, morality, and sentiment of college students, temper their perseverance, and cultivate their will to survive and social adaptability. In addition, in extracurricular activities, college students can also cultivate their excellent personal character according to the characteristics of physical exercise projects. For example, according to the characteristics of sports, we should do a good job in psychological health guidance to correct the mental problems of college students, so as to develop excellent character and morality; or according to the characteristics of sports training items and competition activities, cultivate the competitive will and the spirit of unity, cooperation, and pioneering spirit of college students.

The article "Analysis and Exploration on the Integration of Mental Health Education into College Physical Education Practice" was published in 2022. Journal: Comput Intell Neurosci.

### 5.2. College Physical Education Teaching

With the emphasis of national education on the physical and mental health development of college students, in the newly formulated physical education curriculum standards, sports psychology has become the most important teaching category, and for the first time clearly written into the teaching goals of physical education teaching and physical education courses in colleges and universities. But now, how to reasonably use the psychological teaching resources of modern physical education teaching, find the opportunity of psychological teaching, seize the good opportunity of psychological education, and implement targeted psychological teaching for college students has attracted the attention of more psychological educators. The majority of physical education teachers are gradually deepening the connotation and methods of psychological teaching from teaching practice. For example, in the school sports curriculum, according to the teaching characteristics, cultivate students' psychological emotion of active learning and develop perfect personality; by setting up various interesting extracurricular activities, we can fully mobilize learners' strong thirst for knowledge and cultivate students' psychological feelings of loving reading and activities; use scientific and reasonable training methods to guide students to actively study and train, fully mobilize students' enthusiasm for sports, and cultivate strong interest in sports, so as to fully mobilize students' enthusiasm for learning sports and give full play to their talents. The main connotation of health quality education is to train students' strong will and character by learning sports technology and skills, and fully mobilize the initiative and enthusiasm of college students to exercise.

### 5.3. Campus Sports Culture

The excellent cultural atmosphere of school sports and rich and colorful cultural activities of school sports make students feel comfortable, exhilarated, and full of life. Therefore, actively participating in the construction of a healthy and harmonious school sports and social and cultural environment, and actively participating in the creation of a cultural and educational environment for physical and mental health will greatly promote the school's physical and mental health education. In the construction of school sports civilization, we should conscientiously do a good job in the management of school sports teaching, actively participate in the establishment of sports elective courses, actively participate in the establishment of school sports associations and clubs, arrange school extracurricular physical exercise teaching activities and competitions, and actively participate in the exchange of sports culture between schools, it is the main channel to actively participate in creating an excellent school sports environment. It is the responsibility of every educator to build a campus environment conducive to the physical and mental health development of college students. No matter the school leaders or general administrators, physical education teachers, or principals, they should try their best to build a campus environment conducive to the physical and mental health development of college students. That is, school leaders and administrators should pay attention to the development of campus sports work; physical education teachers should also do well in their own work, actively invest building in and creating a healthy school sports culture, and carry out extracurricular sports activities; the teacher should also actively participate in the construction and be responsible for the extracurricular sports activities of the school class.

The article "Analysis and Exploration on the Integration of Mental Health Education into College Physical Education Practice" was published in 2022. Journal: Comput Intell Neurosci.

## 6. Conclusion and Suggestions

### 6.1. Conclusion

This paper systematically studies the relationship between the physical, physical, mental health knowledge, and psychological level of college students by conducting mental health examinations on 6,000 students from 23 universities, and draws the following conclusions.

1. 24.20% of the research subjects have psychological problems of different degrees, and the positive rate of psychological problems is 10.1%, indicating that the psychological problems of Chinese college students are still serious.
2. The overall average psychological level of college students is changing in the same direction with their physical condition, that is, the physical condition of college graduates is gradually weakening due to the increase of the degree of mental illness.
3. There is a great correlation between college students' sports attitude, activity time, and their physical health level, including three dimensions: students' basic attitude towards sports, time of secondary sports and their adherence to physical exercise, which play a major role.
4. The higher the level of health knowledge structure, the higher the health self-assessment; college students have a higher cognitive structure of their own body, their physical state is better, and their health level is also more higher.
5. In conclusion, the mental health status of college students is closely related to their own physical status and understanding of mental health knowledge. In order to improve the mental health of contemporary college students, it is constructive to integrate mental health education into the practice of physical education in colleges and universities.

### 6.2. Suggestions

1. Build a harmonious mental health knowledge and teaching system, and widely carry out mental health education for college students. Regard the health quality education of college graduates as an organic system, and jointly promote the physical and mental health development of college graduates through the investment of all teachers and mutual cooperation.
2. Create a healthy and harmonious physical education classroom to promote the healthy and harmonious development of college students' body and mind. Using interesting educational methods, through collective teaching activities and overall curriculum, college students are encouraged to actively participate in physical exercise, and a good multilateral communication process is established between teachers and students, so as to create a relaxed and harmonious classroom atmosphere, so that students feel happy from sports, reduce depression, anxiety and bad emotions, and strengthen communication. It not only improves the physique of college students, but also promotes their physical and mental health development.
3. Strengthen the reform of physical education teaching and continuously improve the quality and effect of physical education. Taking the sports programs that college students are most interested in as a carrier, it is integrated into the content of school health education, student physical fitness training, and school sports technology teaching. Through the diversified and vivid sports teaching content, the school sports technology teaching has effectively realized “educating people, sports and hearts.”
4. Opened up a physical education teaching space in colleges and universities and created a body and mind's benign exchange platform for students. It has established an “integrated” college physical education teaching structure inside and outside the curriculum, organically integrated the school sports teaching with extracurricular sports, amateur sports training, and student sports competition. It should expand the time range of the school sports curriculum, and further space for school physical education teaching activities, expand the creating more sports training, and exchange opportunities for college students.

The article "Analysis and Exploration on the Integration of Mental Health Education into College Physical Education Practice" was published in 2022. Journal: Comput Intell Neurosci.

## Figures and Tables

**Table 1:** Analysis of the influence of demographic characteristics on mental health of college students.

Demographic characteristics		Number of persons	Number of psychological disorders	Occurrence rate (%)	X2	*P*
Gender	Male	792	197	24.87	1.455	0.217
	Female	923	218	23.62		

Nation	Han nationality	1614	390	24.16	0.438	0.792
	Minority	101	25	24.75		

Registered permanent residence	Urban residence registration	1183	312	26.37	5.412	0.018

Category	Nonurban household registration	532	103	19.36

Children	Only child	1263	317	25.10	6.374	0.025
Status	Not only child	452	98	21.68		

**Table 2:** Comparison of scores of nine psychological factors between only child and not only child college students.

Psychological factors	Only child	Not only child	*U*	*P*
Somatization	1.42 ± 0.47	1.38 ± 0.41	1.8412	0.2367
Forced	1.84 ± 0.64	1.73 ± 0.59	2.9348	0.0342
Interpersonal relationship	1.91 ± 0.62	1.82 ± 0.67	3.7265	0.0184
Depressed	1.84 ± 0.61	1.66 ± 0.63	4.0148	0.0001
Anxious	1.73 ± 0.54	1.58 ± 0.52	3.5172	0.0024
Hostile	1.77 ± 0.62	1.71 ± 0.58	0.0951	0.8325
Terror	1.48 ± 0.53	1.45 ± 0.51	1.0226	0.2434
Bigotry	1.79 ± 0.62	1.64 ± 0.47	2.1872	0.0285
Psychovenereal disease	1.57 ± 0.55	1.58 ± 0.48	1.1455	0.6018

**Table 3:** List of scores of nine psychological factors of college students of different grades.

Psychological factors	First year in college	Sophomore year	Junior at the university	Fourth year of university
Somatization	1.48 ± 0.53	1.49 ± 0.47	1.46 ± 0.47	1.51 ± 0.50
Force	1.96 ± 0.66	1.84 ± 0.64	1.81 ± 0.59	1.75 ± 0.63
Interpersonal relationship	2.02 ± 0.70	1.93 ± 0.63	1.87 ± 0.63	1.84 ± 0.63
Depressed	1.83 ± 0.66	1.75 ± 0.61	1.79 ± 0.60	1.68 ± 0.60
Anxious	1.71 ± 0.61	1.66 ± 0.55	1.70 ± 0.55	1.72 ± 0.56
Hostile	1.83 ± 0.71	1.78 ± 0.63	1.77 ± 0.64	1.75 ± 0.64
Terror	1.51 ± 0.55	1.48 ± 0.50	1.47 ± 0.51	1.45 ± 0.55
Bigotry	1.77 ± 0.84	1.76 ± 0.60	1.78 ± 0.60	1.70 ± 0.63
Psychovenereal	1.61 ± 0.55	1.65 ± 0.50	1.63 ± 0.52	1.59 ± 0.52

**Table 4:** List of physical condition of college students.

	Height standard weight grade		Vital capacity weight index grade		Grip strength and weight index grade		Standing long jump grade		Bench test score grade		Overall physique evaluation grade	
	Number of persons	Percentage	Number of persons	Percentage	Number of persons	Percentage	Number of persons	Percentage	Number of persons	Percentage	Number of persons	Percentage
Excellent (normal)	515	30.03%	191	11.14%	875	51.02%	35	2.04%	221	12.89%	154	8.98%
Good (low)	1028	59.94%	411	23.97%	549	32.01%	231	13.47%	726	42.33%	738	43.03&
Pass	—		686	40%	206	12.01%	694	40.47%	664	38.72%	771	44.96%
Pass	172	10.03%	427	24.09%	85	4.96%	755	44.02%	104	6.06%	52	3.03&

The article "Analysis and Exploration on the Integration of Mental Health Education into College Physical Education Practice" was published in 2022. Journal: Comput Intell Neurosci.

**Table 5:** Comparison of six physical fitness indexes of college students with different mental health levels.

Physical index score	Normal group	Mild group	Moderate group	Severe group	*F*	Sig
Total physical fitness score	77.4 ± 4.74	77.1 ± 7.12	74.7 ± 6.17	72.4 ± 8.89	3.49	0.018
Height standard weight score	10.47 ± 2.71	10.55 ± 2.92	10.43 ± 2.65	9.23 ± 2.22	1.65	0.181
Bench test score	16.87 ± 1.97	16.50 ± 2.31	16.16 ± 1.82	15.23 ± 2.29	3.28	0.023
Vital capacity body mass index	12.23 ± 2.11	11.26 ± 1.79	11.06 ± 1.74	10.80 ± 2.04	3.14	0.028
Standing long jump score	21.30 ± 2.94	19.83 ± 2.37	18.63 ± 1.77	17.20 ± 2.42	15.60	0.000
Grip strength body mass score	18.67 ± 2.08	18.63 ± 1.77	17.20 ± 2.42	17.96 ± 2.48	2.93	0.037

**Table 6:** Comparison of nine mental health factors of college students with different physical conditions.

Mental health factors	Excellent physique group	Good constitution group	Physical fitness passing group	Physical fitness unpassed group	*F*	*P*
Somatization	1.38 ± 0.41	1.42 ± 0.47	1.53 ± 0.47	1.82 ± 0.46	16.71	0.0001
Forced	1.79 ± 0.59	1.84 ± 0.64	1.89 ± 0.60	2.10 ± 0.63	15.16	0.0001
Interpersonal relationship	1.65 ± 0.67	1.89 ± 0.62	1.92 ± 0.67	2.08 ± 0.68	16.06	0.0001
Depressed	1.56 ± 0.63	1.74 ± 0.61	1.79 ± 0.61	1.92 ± 0.66	16.91	0.0001
Anxious	1.58 ± 0.52	1.73 ± 0.54	1.75 ± 0.57	1.91 ± 0.65	18.34	0.0001
Hostile	1.68 ± 0.58	1.71 ± 0.62	1.77 ± 0.70	1.98 ± 0.69	20.25	0.0001
Terror	1.43 ± 0.51	1.45 ± 0.53	1.45 ± 0.48	1.61 ± 0.66	12.53	0.0001
Bigotry	1.49 ± 0.47	1.62 ± 0.62	1.67 ± 0.63	1.90 ± 0.54	14.81	0.0001
Psychovenereal	1.48 ± 0.48	1.47 ± 0.55	1.63 ± 0.51	1.94 ± 0.36	15.37	0.0001

## Data Availability

The experimental data used to support the findings of this study are available from the corresponding author upon request.
